# Biomechanics of Volleyball Players' Run-Up and Take-Off Link under Deep Learning

This article has been retracted.

**DOI:** 10.1155/2022/8409626

**Published:** 2022-07-14

**Authors:** Lejun Hu, Lantao Liu, Kai Zhao

**Affiliations:** ^1^Zhejiang Sci-Tech University, Hangzhou 310000, Zhejiang, China; ^2^Department of Physical Education, Central South University, Changsha 410083, China; ^3^China Volleyball College, Beijing Sport University, Beijing 100089, China

## Abstract

In volleyball, the correct approach and start (including the number of steps and stride speed) are a prerequisite for all technical movements to attack. It can not only improve the horizontal speed of the athlete, but also properly convert the total speed into vertical speed, so that the hitting point is improved and the ball speed is accelerated. To explore the biomechanical characteristics of lower limb movements in the run-up and take-off stage of volleyball spiking, this paper takes four male volleyball players from the Physical Education College of X University as the research objects to analyze the kinematics and dynamics of the run-up process and the take-off process. This paper uses the precise recognition method under the background of deep learning to accurately capture the movements of the research object. This paper discusses the effects of time, speed, distance, knee, and hip parameters (angle, joint muscle torque, and power) on the effect of spiking techniques. It is expected to provide reference for the diagnosis, guidance, and muscle strength training of this special technical movement. The  research results show that the horizontal speed of No. 2 athlete is 3.62 m/s and the vertical speed is 2.71 m/s when he takes off. The  landing time is 0.375 s and the lift-off time is 0.16 s. The torque and power of the knee joint changed greatly during the take-off process, and the change of the hip joint was small.

## 1. Introduction

Spike is an important scoring method in volleyball. With the height of volleyball players, the level of jumping is getting higher and higher. To improve the effect of spiking, the players' offensive strategy has gradually changed from a flat attack to a three-dimensional attack. The techniques of front row spiking, front row coping, and backcourt spiking have been integrated, increasing the difficulty of the opponent's interception. In volleyball, the technical action of spiking is divided into four processes: run-up, take-off, air, and landing. Among these four processes, the run-up process and the take-off process are the most important. The effect of running and jumping on both feet directly determines the success rate and quality of technical and tactical actions such as blocking and spiking. There are also a large number of experts and scholars who have carried out kinematics and dynamics analysis and research on the various phases of the double-foot approach and take-off action. Some foreign studies are also trying to establish the action model of the human vertical jump, but the gap between scientific research and training practice still needs to be filled little by little. This article is based on the start-up stage of a complete spiking action, which lasts only 0.6 seconds. It is the basic stage of the entire spiking action. In this stage, if there are some unreasonable and unstable movements, it will greatly affect the subsequent technical movements such as flying, blocking, and spiking.

Deep learning is an important branch of machine learning. Unlike algorithms that involve specific tasks, it is based on the learning of representations from the data. Deep learning simulates the neural network model of the human brain, which uses multilevel nonlinear operation units in series to extract and transform data information. Each sequence takes the output of the previous sequence as input, and it takes the initial data as the input of the first sequence to obtain the final feature information. Deep learning technologies such as deep neural networks, convolutional neural networks, and recurrent neural networks have been widely used in computer vision, speech recognition, natural language processing, audio recognition, social networks, and other fields. In this paper, through the method of high-speed camera video acquisition, the accurate recognition algorithm in artificial neural network is used. It collects data on the running width, the running distance, and the dynamic change process of the knee and hip joints in the run-up and take-off stage. This paper analyzes joint muscle torque and power. Through the kinematic analysis of the run-up process and the dynamic analysis of the take-off process, this paper determines the functions and characteristics of the knee joint and the hip joint in the run-up and take-off process. It can diagnose the movement situation and have a better grasp of the dynamic changes of each joint. The purpose of this paper is to investigate the biomechanical properties of the volleyball spike during the approach and take-off process to better understand the movement characteristics and muscle activity of the technique.

## 2. Related Work

In recent years, researchers from various countries have discussed the application and development prospects of deep learning methods in various fields. It has done relevant research in all aspects and applications of deep learning methods. Chen et al. combined the idea of deep learning with the classification of hyperspectral data. They also proposed a new deep learning framework to fuse two classification methods (spectral information-based classification and spatial-dominant information-based classification) for maximum recognition precision. They proposed a method based on principal component analysis, deep learning, and logistic multivariate regression model. It is demonstrated that the classifier constructed on this basis has better performance [1]. Kermany et al. have developed a deep learning-based medical diagnostic to screen patients with retinopathy. The framework uses artificial neural network technology based on transfer learning, which has been widely used in optical coherence tomography images. Experiments have confirmed that this method can accelerate the diagnosis of retinopathy, and it can promote its early treatment and improve its clinical efficacy [2]. Lee discussed the development and implementation of blockchain technology in cyber-physical production systems. He proposed a unified three-tier blockchain architecture as a guideline for the industry. It clearly identifies the potential of blockchain. It aimed to integrate and synchronize the world of machines and manufacturing facilities into the networked computing space to move towards Industry 4.0 [3]. Oshea and Hoydis presented and discussed several new implementations of deep learning at the physical level. In the process of autocoding communication systems, they developed a new approach that views the design of a communication system as an end-to-end reconfiguration, with a single process that optimizes both transmitting and receiving elements. Based on this, they applied it to networks with multiple senders and receivers and introduced it into machine learning models [4]. Ravi et al. presented a comprehensive overview of relevant research on the use of deep learning in health informatics. They provided an insight into the relevant advantages, potential pitfalls, and prospects. They focused on the application of deep learning in bioinformatics, medical imaging, universal sensing, medical informatics, and public health [5]. Schirrmeister et al. have developed convolutional neural network-based electroencephalopathological decoding technology and visualized deep learning techniques. They performed an analysis of pathological and normal EEGs from the abnormal EEG corpus at Temple University School of Medicine. On the basis of CNN, they used two CNN architectures to decode tasks in electroencephalopathology. Results showed that convolutional neural networks were 6% more accurate than the published results for this dataset when decoding EEG pathology [6].

## 3. Artificial  Neural  Networks  and Convolutional Neural Networks

### 3.1. Artificial Neural Network

Artificial neural network is formed based on the neural network in the human brain. After a lot of anatomical research, scientists gradually understand the composition principle of neural networks. It has two advantages: first, each branch is parallel and does not interfere with each other. Second, the neural network has good learning and generalization ability. During training, reasonable outputs are obtained even without learning. These two advantages of the neural network enable the neural network to simulate the relationship between complex functions, and it can use the learning method to find the approximate solution of the function [7]. In the brain, nerve cells transmit information through chemical information, and computers can use binaries to simulate chemical information in cells. Usually, to facilitate simulation, neurons in the brain are usually divided into two states: excitation and inhibition, 1 for excitation and 0 for inhibition [8]. The excitatory and inhibitory signals of a neuron are influenced by the dendrites of that neuron, which can receive stimulation signals from multiple neurons simultaneously. And through a series of complex operations, it finally forms a specific excited or inhibited state.

Machine learning is a sure-fire way to artificial intelligence, and it encompasses knowledge from many disciplines. Fundamentally speaking, machine learning is to extract the statistical rules of the learned objects from the massive training samples. It enables human beings to “cognize” and correctly predict new things [9]. Before the advent of deep learning, many traditional machine learning methods have been well applied. However, for some complex problems or problems with nonlinear properties, it is often difficult to classify them with traditional machine learning methods. The extracted features are summed up by a large amount of research experience, and the processing of the same problem is also very complex and unstable, and these are determined by the large amount of experience of scientific researchers. However, deep learning does not require human intervention; just throw a large amount of data to it, and it can learn autonomously. The principle of artificial neural network is to simulate the activity of neurons in the human brain, and it is expected to establish a model that can learn autonomously. Since its emergence, neural networks have good potential for nonlinear regression and classification decisions. However, it requires a large number of samples, and the amount of computation involved is also very large, and it is prone to local optima during the training process, which makes the generalization ability of the neural network poor [10]. However, with the rapid development of information technology and the rapid development of computer hardware, the computing power of computers has been greatly developed. And the training algorithm has also been continuously updated, and people's understanding of deep neural networks is constantly developing and improving.

Figure 1 shows the perception mechanism of a single neuron. It, like neurons in the human brain, has two different output modes. The perceptron is the most basic model in the feedforward network. After receiving the input signal, it is weighted with the corresponding weights, and then the final output is obtained by the activation function.

In the perceptron model diagram, *x*_1_, *x*_2_,…, *x*_*n*_ are the input data, and *w*_1_, *w*_2_,…, *w*_*n*_ are the corresponding weights. The specific calculation formula is as follows:

(1) $$\begin{array}{c} y=\alpha \left(\sum_{i=1}^{n}w_{i}x_{i}+b\right). \end{array}$$

In this model, *α*( ) is the activation function, *b* is the bias, and the learning process of the neuron is to adjust the weight parameter *W*, so that the output of the training sample is the closest to the actual value. However, the perceptron model is only suitable for decomposable linear problems, while the artificial neural network is a multilayer perceptual system composed of one or more neurons, and the output of the neurons in the previous layer is provided to the neurons in the next layer. An artificial neural network is a multilayered perceptron, each of which contains one or more neurons, and the output of the neurons in the previous layer is the input of the neurons in the next layer. When the number of neurons is sufficient, it can approximate any complex continuous functions and logical expressions, so that the artificial neural network has better representation ability [11].

The artificial intelligence network model is consistent with a three-stream system consisting of an input layer, a hidden layer, and a producer layer. The input layer is the gateway to the entire network object. Sample data enters the network template through this layer and it is exported to the hidden layer. The hidden layer contains one or more layers of neurons. The more the layers, the stronger the representation ability of the neural network, but the corresponding training difficulty will also increase.  Figure 2 is an artificial neural network model with only one hidden layer. The output layer is the final output of the neural network, which is generally the classification result.

A neural network is a way to model the relationship between input data and target data. Through shallow neural network to explore the correlation between input data and actual output, the neural network can only obtain a simple functional relationship with the target data. However, more complex relationships cannot be obtained [12]. Moreover, the more the hidden layers in the neural network are, the more abstract the feature information will be. It enables the neural network to better simulate more complex functional relationships from the initial linear relationship to the subsequent nonlinear functions.

### 3.2. Backpropagation Algorithm

Backpropagation algorithm is a learning algorithm in the field of artificial intelligence, which is a typical neural network learning algorithm. The basic idea of this method is as follows: in the process of neural network training, the output error of each level will be backpropagated to the neural network. The neural network will correct the weight and bias of the network according to the feedback error to reduce the deviation from the target data and make it closer to the target data. In the training process of the neural network, it adopts the gradient descent algorithm. Its function is to correct weights and bias by learning the training set [13].

The formula principle of the backpropagation algorithm is as follows.

*w*_*jk*_^*l*^ represents the connection weight between the *j*th neuron in the *l*th layer and the *k*th neuron in the previous layer. *b*_*j*_^*l*^ represents the bias of the *j*th neuron in the lth layer; *z*_*j*_^*l*^ represents the input of the *j*th neuron in the *l*th layer. The output value can be expressed as

(2) $$\begin{array}{c} a_{j}^{l}=\delta \left(\sum_{k}w_{jk}^{l}a_{k}^{l-1}+b_{j}^{l}\right), \end{array}$$

where *δ* represents the activation function.

The cost function is used to measure the gap between the predicted value and the actual value. The purpose of the training is to reduce the output of the cost function step by step, so that the output of the network is closer and closer to the actual value. Usually, a quadratic cost function or its variant is used as the cost function:

(3) $$\begin{array}{c} C=\frac{1}{2n}{\sum_{x}\left\|y\left(x\right)-a^{L}\left(x\right)\right\|}^{2}. \end{array}$$

Among them, *x* represents the input sample, *y* represents the actual classification, *a*^*L*^ is the network output, and *L* is the number of network layers.

The formula for calculating the error generated by a neuron is

(4) $$\begin{array}{c} \delta_{j}^{l}=\frac{\partial C}{\partial z_{j}^{l}}. \end{array}$$

The output of the cost function is

(5) $$\begin{array}{c} C=\frac{1}{2}{\left\|y-a^{L}\right\|}^{2}=\frac{1}{2}{\sum_{j}\left(y_{j}-a_{j}^{L}\right)}^{2}. \end{array}$$

The output error of the network is

(6) $$\begin{array}{c} \delta^{L}=\nabla_{a}C•\delta^{\prime }\left(z^{L}\right). \end{array}$$

Among them, ∙ is the multiplication between matrices.

The derivation process of formula (6) is as follows:

(7) $$\begin{array}{c} \delta_{j}^{L}=\frac{\partial C}{\partial z_{j}^{L}}=\frac{\partial C}{\partial a_{j}^{L}}\cdot \frac{\partial a_{j}^{L}}{\partial z_{j}^{L}},\\ \delta^{L}=\frac{\partial C}{\partial a^{L}}•\frac{\partial a^{L}}{\partial z^{L}},\\ =\nabla_{a}C•\delta^{\prime }\left(z^{L}\right). \end{array}$$

Calculating the errors in each layer of the network at once:

(8) $$\begin{array}{c} \delta^{l}=\left({\left(w^{l+1}\right)}^{T}\delta^{l+1}\right)•\delta^{\prime }\left(z^{l}\right). \end{array}$$

The derivation process of formula (8) is as follows:

(9) $$\begin{array}{c} \delta^{l}=\frac{\partial C}{\partial z_{j}^{l}}=\sum_{k}\frac{\partial C}{\partial z_{k}^{l+1}}\cdot \frac{\partial z_{k}^{l+1}}{\partial a_{j}^{l}}\cdot \frac{\partial a_{j}^{l}}{\partial z_{j}^{l}},\\ \delta^{l}=\sum_{k}\delta_{k}^{l+1}\cdot w_{k}^{l+1}\cdot \delta^{\prime }\left(z_{j}^{l}\right),\\ =\left({\left(w^{l+1}\right)}^{T}\delta^{l+1}\right)•\delta^{\prime }\left(z_{j}^{l}\right). \end{array}$$

Calculating the weight gradient:

(10) $$\begin{array}{c} \frac{\partial C}{\partial w_{jk}^{l}}=\delta_{j}^{l}\cdot \frac{\partial \left(w_{jk}^{l}a_{k}^{l-1}+b_{j}^{l}\right)}{\partial w_{jk}^{l}}=a_{k}^{l-1}\delta_{j}^{l}. \end{array}$$

Calculating the bias gradient:

(11) $$\begin{array}{c} \frac{\partial C}{\partial b_{j}^{l}}=\delta_{j}^{l}\cdot \frac{\partial \left(w_{jk}^{l}a_{k}^{l-1}+b_{j}^{l}\right)}{\partial b_{j}^{l}}=\delta_{j}^{l}. \end{array}$$

Therefore, the steps of the backpropagation algorithm are as follows:

(a) Input training set.
(b) For each sample *X* in the training set, set the activation value corresponding to the input layer to *a*^*l*^.
Forward propagation:
  (12) $$\begin{array}{c} z^{l}=w^{l}a^{l-1}+b^{l},a^{l}=\delta \left(z^{l}\right). \end{array}$$
(c) Calculating error generated by the output layer:
  (13) $$\begin{array}{c} \delta^{L}=\nabla_{a}C•\delta^{\prime }\left(z^{L}\right). \end{array}$$
(d) Calculating the backpropagation error:
  (14) $$\begin{array}{c} \delta^{l}=\left({\left(w^{l+1}\right)}^{T}\delta^{l+1}\right)•\delta^{\prime }\left(z^{l}\right). \end{array}$$
(e) Gradient descent training parameters:
  (15) $$\begin{array}{c} w^{l}⟶w^{l}-\frac{\eta }{m}\sum_{x}\delta^{x,l}{\left(a^{x,l-1}\right)}^{T},\\ b^{l}⟶b^{l}-\frac{\eta }{m}\sum_{x}\delta^{x,l}. \end{array}$$

### 3.3. Convolutional Neural Networks

The cumulative neural network is a new neural network based on the synthetic neural network. By doing integration work on it, it has much better compatibility than the virtual network. Compared with artificial intelligence networks, the advantages of networked networks are as follows.

#### 3.3.1. Local Connection

Modern biology believes that the picture seen by the human eye is from the part of the whole. In an image, the closer the pixels are spaced, the tighter they are connected and vice versa. Therefore, each node only needs to be connected to a local area in the image and does not need to be fully connected to the features of the previous level. In convolutional neural networks, local connections reduce the number of parameters needed in the learning process. In a convolutional neural network, the local connection is to combine the neurons of this layer with the neurons of the upper layer, thereby reducing the parameters required in the learning process. Due to the large number of parameters in the network, the training of the network becomes more difficult. Therefore, the method of local connection is an important factor in the evolution of artificial neural networks from shallow to deep neural networks [14].

#### 3.3.2. Weight Sharing

Compared with the full connection, the partial connection can greatly reduce the number of parameters, but, in the case of a large number of features, even if the partial connection is used, it will cause a large amount of parameters [15]. Convolution is a method to extract features from an image; however, feature extraction should be position independent. That is, using the convolution check image to perform convolution (feature extraction), the same feature should be extracted, which is weight sharing.

#### 3.3.3. Pooling

By extracting the features of the convolutional layer, the feature map of part of the original image can be obtained, but, due to its large size, it cannot be directly classified. Since there is a large correlation between adjacent pixels in the image, the bottom-shaped parts and adjacent pixels are replaced with the same resolution without much loss of detail. It created a feature map using the method; by this way, a new feature map was obtained. This process is called “aggregation” [16]. Pooling can also improve the build performance and strength of the network, and it can prevent the network from running efficiently.

#### 3.3.4. Multiple Convolutional Layers

As the number of network layers increases, the obtained image features will become more reasonable, so using multiple convolutional layers for image feature extraction can achieve better fitting effects [17].

The lexical network can effectively reduce the amount of space required for network training and reduce the amount of data required for network training, thus improving the network training efficiency. In the convolutional neural network, the essence of weight sharing is to use a specific area in the same convolutional check image to perform convolution operations, so that the same feature information can be extracted from different positions. Therefore, even after the image has been translated, the convolutional neural network can still recognize the image. It does not affect the feature extraction of convolutional neural networks due to image movement [18, 19].

As shown in Figure 3, the hard core is a multilayer network, which is consisted by a layer input, a convolutional layer, a downsampled layer (i.e., layer aggregation), a fully connected layer, and a layer output. In a complex network, signals are transmitted sequentially by many neuronal nodes. It then uses continuous convolution pooling techniques to decode, deduce, and pool to map the signal to the feature space of the hidden layer and classify the output [20].

*(1) Convolutional Layer*. Convolutional layers essentially use filtering operations to complete local feature responses. The convolution kernel is a middle filter, which uses the same convolution kernel to scan the entire image and extract all features, to achieve the purpose of weight sharing. Usually, each convolution layer has several convolution kernels, the image features extracted from these convolution kernels are called feature maps, and the calculation formula is as follows:

(16) $$\begin{array}{c} y_{j}^{l}=\alpha \left(\sum_{i=1}^{N_{j}^{l-1}}w_{j}⊗x_{i}^{l-1}+b_{j}^{l}\right),j=1,2\ldots M. \end{array}$$

Among them, *y*_*j*_^*l*^ is the bias value, *N*_*j*−1_^*l*^ is the feature quantity of each feature map, *M* is the feature quantity of each convolutional layer, and *α*( ) is the activation function. Each feature map can only represent one type of feature, and the later convolution layer actually obtains more expressive features by continuously extracting the underlying feature map. Therefore, when increasingly abstract features are obtained, the number of feature maps in the network layer will increase accordingly.

*(2) Pooling Layer*. The feature information after the convolution layer convolution is still very large, which will not only bring about the decline of the computing performance, but also cause the phenomenon of overfitting. Therefore, while reducing the feature dimension, it can extract representative feature information and make the processed feature map have a larger receptive field. This operation of replacing the whole feature with partial features is called pooling operation. The pooled image still has translation invariance, and the pooling operation will blur the specific position of the feature. After the image is translated, the same feature can still be generated. The pooling operation can further abstract the features of a local area, an element in the pooling corresponds to a region in the input data, and the pooling effect can reduce the number of parameters and reduce the image dimension [21].

Common loading methods include maximum load and average load. The maximum concentration is to choose the maximum value in each subregion as the final result. And choose the mean of all the values as the final result.  Figure 4 shows a schematic diagram of two pooling effects with a pooling step size of 2.

*(3) Fully Connected Layer*. In a traditional multilayer perceptron, a fully connected layer is a hidden layer similar to a multilayer perceptron. The convolutional neural network is a neural network in which each layer of neurons is connected to the neurons of the next layer. In the convolutional neural network, the specific calculation formula of the fully connected layer is as follows:

(17) $$\begin{array}{c} h_{W,b}\left(x\right)=\alpha \left(W^{T}x\right)=\alpha \left(\sum_{i=1}^{3}W_{i}x_{i}+b\right), \end{array}$$

where *h*_*W, b*_(*x*) represents the output of the fully connected layer; *x*_*i*_ represents the output of the previous layer of neurons, that is, the input of the fully connected layer; *W*_*i*_ represents the weight of the connection between neurons; *b* represents the bias.

Allowing complex neural networks to compare more complex business relationships, implementations are often integrated behind a complex layer or a fully connected layer. It allows difficult networks to learn stronger working relationships. In addition, adding deployment functionality to a complex network can add unnecessary components to the network. It allows complex neural networks to perform any unusual function, which increases the ability of neural networks of solving behavioral problems. Popular deployment services include ReLU deployment service, Sigmoid deployment service, and Tanh deployment service [22]. The formulas are as follows:

(18) $$\begin{array}{c} f\left(x\right)=\max\left(0,x\right),\\ f\left(x\right)=\frac{1}{1+e^{-x}},\\ f\left(x\right)=\frac{e^{x}-e^{-x}}{e^{x}+e^{-x}}. \end{array}$$

The image of the sigmoid deployment function is a sigmoid regression, so the sigmoid deployment function is also known as the sigmoid function. Because the sigmoid activation function is continuous and monotonic between (0, 1) and the output range of the function is limited, the sigmoid activation function is often used in binary classification problems. The image of the sigmoid deployment function is shown in Figure 5.

The image of the Tanh activation function is a hyperbola, so the Tanh activation function is also called the bitangent function. The advantage of the Tanh activation function is that it works well in scenes with significantly different feature information, and it expands the feature effect during training.

The ReLU activation function is a nonsaturating activation function, also known as a rectified linear unit. Compared with the most commonly used deployment services, the ReLU deployment function has strong offline ReLU deployment capabilities in the network. For faulty performance in the network, the ReLU implementation function can keep the model's integration rate at a relatively constant level. Therefore, the ReLU deployment function is also a frequently used deployment service in virtual networks.  Figure 6 is a function image of ReLU.

## 4. Experiment of Volleyball Approach and Jump

The research objects of this paper are 4 male volleyball players from the Physical Education College of X University, all of whom have reached the national second level and above. The subjects did not perform high-intensity training or competition one week before the experiment, and the subjects were in good physical condition on the test day. The basic information of the experimental subjects is shown in Table 1.

This paper takes the spiking action of volleyball as the research content and compares and analyzes two typical actions represented by front row No. 4 and back row No. 6. This paper focuses on the analysis of the kinematics and dynamics parameters of the two stages of the spiking run-up process and the take-off process.

### 4.1. Kinematics of Approach Process

The run-up process refers to the process from the start of the first step to the moment when both feet touch the ground. To approach the ball and choose the jumping point, the human body should be given a suitable and faster movement speed according to the goals of different projects before jumping. It also prepares the body for the best take-off position. One of the purposes of the run-up is to prepare for take-off and hitting the ball, and the other is to obtain a greater horizontal speed. According to the theory of sports anatomy, when the athlete's take-off leg support strength reaches a certain level, the faster the run-up speed, the greater the impact on the take-off leg strength. The muscle load of the take-off leg will also increase accordingly, and the extensor muscles of the take-off leg will also adjust as many muscle fibers as possible, so that the muscle contraction force is greatly improved. Therefore, the maximum approach speed is very critical to the height of the jump.  Table 2 shows the stride length, approach distance, and maximum speed of the test subjects in the run-up stage.

The experimental subjects all adopted a three-step approach. During the approach, the approach width gradually increased, and the last step reached the maximum. The average approach distance was 3.30 m, and the maximum approach speed during the approach was 4.35 m/s. And the research subjects' run-up showed that the first step was small, the second step was large, the stride gradually increased, and the second step had the largest stride, accounting for 52% of the approach distance. Athlete No. 1 has the largest stride in the second step, 1.89 m, the first step is 0.93 m, the second step is 0.83 m, and his approach speed is 4.54 m/s. The second and first steps of No. 2 athlete were both 1.56 m and 1.03 m smaller than those of No. 1 athlete. However, its parallel stride is greater than that of No. 1 athlete, which is 0.91 m, and its approach speed is 4.67 m/s. It can be concluded that the stride length also affects the approach speed. In addition, the parallel distances of the study subjects varied widely. And there is a significant positive correlation between parallel stride and approach speed. Technically speaking, the athlete must first observe the angle and arc of the ball to determine the landing point and then determine the direction and time of the take-off. Therefore, in the run-up phase, the first step should not be too large. The second step has a large stride. One is to lower the center of gravity and convert the inertial force after braking into an upward speed. The second is to ensure the position of the jump and the accurate landing point after the start. As the approach speed increases, so does the parallel distance. If the step distance is too short, the lateral speed buffer cannot be fully completed, so that the forward thrust after the jump is large and it is easy to fall.

### 4.2. Dynamic of Take-Off Process

Taking off is a prerequisite for offensive serving and spiking. Its purpose is to gain height and to choose the right timing. The correct take-off method includes both height and distance. Height: jumping higher at a given distance not only increases the angle of the ball over the net, but also gives enough time to ensure a rotating swing. Distance: the longer the jump is, the more power the body gets. It can not only prolong the hitting distance at the moment of hitting the ball, but also increase the impact on the ball, making the hitting speed faster and the attacking power stronger. At the same time, the increase of the jumping distance reduces the interval between the hitting point and the landing point. At the same speed, it reduces the time in which the ball is in the air, making it more difficult for the opponent to catch the ball. The increased jumping distance allows players to quickly return to their position on the field, either defensively or offensively.

Table 3 shows the lift-off angle of the center of gravity and the loss rate of horizontal velocity during the take-off stage.

Through the experimental research on the center of gravity speed and the take-off time of each athlete during the take-off process, this paper analyzes the dynamics of the athletes during the take-off process. It includes the following aspects: horizontal speed, vertical speed, landing time, and time off the ground. The research results are shown in Figures 7 and 8, respectively.

As can be seen from Figure 7, the horizontal speed of No. 4 athlete is small (2.44 m/s), but his vertical speed is high (2.93 m/s), which is an upward vertical jump. Athletes No. 1 and No. 2 had higher horizontal speeds when they took off 3.3 m/s and 3.62 m/s, respectively, while their vertical speeds were relatively small (2.65 m/s, 2.71 m/s), showing an obvious forward rush. Among them, athlete No. 2 obtained a larger vertical speed when he took off, which indicated that athlete No. 2 had a reasonable take-off action. It is not only conducive to maintain a horizontal forward thrust, but also conducive to the vertical rise of the center of gravity. After taking off, the center of gravity can obtain the appropriate height and distance. In the case of a certain take-off speed, the higher the horizontal speed is, the more favorable it is to rush forward and obtain a suitable distance. The higher the vertical speed, the better the outcome for jumping and getting a suitable height.

Landing time refers to the difference in the time between the landing of the right foot and the landing of the left foot during the run-up process. It is an important indicator to measure the time of the single support of the right foot. The time off the ground refers to the time difference between the left foot and the moment when the left foot leaves the ground. It is used to measure the time of the left foot single support. It can be seen from Figure 8 that athlete No. 4 has a short time off the ground (0.12 s) and the single support time of the left foot is short, showing the movement state of the left and right feet leaving the ground almost at the same time. Athletes 1 and 2 were off the ground longer than athletes 3 and 4. That is, athletes Nos. 1 and 2 support the left and right feet longer than athletes Nos. 3 and 4. This shows that the landing and lifting of the left and right legs are in order during the spiking take-off. Athlete No. 2 has the largest difference in landing time, with both feet landing on the ground in turn and the right foot ahead of the left, which meets the mechanical requirements of jumping. Judging from the take-off and landing time, athlete No. 4 took 0.2 s and took the shortest time, and athlete No. 2 took 0.345 s as the longest jump. The length of time is closely related to the size of the study object and the size of the step. The shorter the distance between the feet is, the shorter the take-off time is, and the faster the take-off action is completed. To a certain extent, the take-off time can reflect the range of buffering and kicking during the take-off stage.

Through the data collection of 4 athletes, the angle changes of the knee and hip joints were studied, and the average test data of these four athletes were summarized and tabulated, as shown in Table 4.

Since the joint muscle moments of the knee and hip joints of the 4 players are similar to the power curves when the volleyball spike takes off, only player 2 is used for analysis, as shown in Figures 9 and 10.

It can be seen from Figure 9 that athlete No. 2 reaches the maximum knee joint muscle torque (0.38 N∙m) at 0.45 s and the hip joint muscle torque reaches the maximum value (0.22 N∙m) at 0.25 s. From 0 to 0.25 s, the knee joint muscle torque increased significantly, while the hip joint muscle torque increased gently. At 0.25∼0.35 s, the knee joint muscle torque continued to increase, while the hip joint muscle torque began to decrease. At 0.35∼0.45 s, the knee joint muscle torque basically remained between 0.36 and 0.38, and the hip joint muscle torque slowly decreased. From 0.45 to 0.60 s, the knee joint muscle torque decreased from 0.38 N∙m to 0.03 N∙m, and the hip joint muscle torque decreased from 0.14 N∙m to −0.03 N∙m.

It can be seen from Figure 10 that the knee joint muscle power of No. 2 athlete reached the maximum value (2.28 W) at 0.45 s. From 0 to 0.25 s, the knee muscle power changed from a positive value to a negative value, from 0.05 W centripetal to 2.12 W eccentric. At 0.25∼0.35 s, the eccentric power of knee joint muscles gradually decreased, and, at 0.35 s, the eccentric power decreased to 0. From 0.35 to 0.45 s, the concentric power of the knee muscles gradually increased, and the concentric power reached the maximum value at 0.45 s. From 0.45 to 0.60 s, the centripetal power of the knee joint muscle decreased continuously to 0.01 W. Athlete No. 2 showed less significant changes in hip muscle power compared to knee muscle power. From 0 to 0.25 s, the eccentric power of the hip muscles basically was maintained between 0.1 and 0.2 W, and, from 0.25 to 0.60 s, the centripetal power of the hip muscles first slowly increased to 0.5 W and then decreased to 0.

## 5. Discussion

1. The whole approach run process showed that the first step was small, the second step was large, and the stride gradually increased. The second step has the largest amplitude, accounting for 52% of the total run-up distance, and the maximum speed of the run-up is also generated in this step. In this way, the runner can gradually increase the speed of the center of gravity to facilitate the transition between the two steps.
2. The moment and power of the knee joint have great changes during the take-off process. Small changes in the hip joint are not conducive to the full use of the hip extensor group, which may lead to poor take-off height. It is recommended to attach importance to the training of hip extension in the approach and take-off training and appropriately increase the range of motion of the hip joint and the contribution rate during the take-off process.

## 6. Conclusion

The experimental part of this paper mainly studies the change trend of the running width, distance and speed, knee joint and hip joint muscle torque, and power of male volleyball players in the run-up and take-off link, but there are also some limitations. First, the sample size is too small, which cannot reflect the general laws and development trends of volleyball players in the run-up and take-off link. Therefore, this article is only a small case study. It is recommended to do further generalization and test in future research to get the final conclusion. Second, although this paper focuses on the change trend of the knee and hip joints of volleyball players during the run-up and take-off, the experiment is slightly one-sided in the absence of the change trend of the ankle joint angle. It is recommended that subsequent researchers try to add ankle joint indicators to qualitatively and comprehensively discover relevant laws and characteristics.

## Figures and Tables

**Figure 1:** Schematic diagram of the neuron perceptron model.

**Figure 2:** Schematic diagram of a single hidden layer neural network.

**Figure 3:** Convolutional neural network structure diagram.

**Figure 4:** Schematic diagram of two pooling effects.

**Figure 5:** Sigmoid function image.

**Figure 6:** ReLu function image.

**Figure 7:** Speed comparison chart of take-off stage. Figure 7 (a) shows the horizontal speed of each athlete during the take-off process. Figure 7 (b) shows the vertical speed of each athlete during the take-off process.

**Figure 8:** Time comparison chart of take-off stage. Figure 8 (a) shows the landing time of each athlete during the take-off process. Figure 8 (b) shows the time off the ground for each athlete during the take-off process.

**Figure 9:** Muscle moments of the knee and hip joints. Figure 9 (a) shows the knee joint muscle torque during the take-off of No. 2 athlete. Figure 9 (b) shows the hip joint muscle moment during the take-off of No. 2 athlete.

**Figure 10:** Muscle power of the knee and hip joints. Figure 10 (a) shows the knee joint muscle power during the take-off of No. 2 athlete. Figure 10 (b) shows the power of the hip joint muscles of No. 2 athlete during the take-off process.

**Table 1:** Basic body shape indexes of subjects.

Number	Height (m)	Weight (kg)	Age	Sports level
1	1.92	86	23	Level 1
2	1.88	89	21	Level 2
3	1.90	90	22	Level 2
4	1.87	78	23	Level 2

**Table 2:** Running width and speed data table.

Number	Width (m)			Distance (m)	Speed (m/s)
	First step	Second step	Parallel step		
1	0.93	1.89	0.83	3.65	4.54
2	1.03	1.56	0.91	3.50	4.67
3	0.67	1.67	0.76	3.10	4.23
4	0.61	1.59	0.77	2.97	3.98

**Table 3:** Lifting angle of center of gravity and loss rate of horizontal speed in take-off stage.

Number	Horizontal speed loss (%)	Lifting angle of gravity center (°)
1	27.32	47
2	22.48	42
3	38.8	50
4	43.7	55

**Table 4:** Knee and hip joint angles at different times.

Time (%)	Knee angle (°)	Hip angle (°)
5	149.35	118.09
10	140.56	123.30
15	132.73	122.14
20	126.68	116.62
25	120.89	121.31
30	110.69	129.52
35	107.38	138.69
40	115.74	143.42
45	122.25	144.35
50	129.00	148.92
55	145.73	152.34
60	139.20	158.83

## Data Availability

The data underlying the results presented in the study are available within the article.

## References

[1] Chen Y., Lin Z., Zhao X., Wang G., Gu Y. (2014). Deep learning-based classification of hyperspectral data. *Ieee Journal of Selected Topics in Applied Earth Observations and Remote Sensing*.

[2] Kermany D. S., Goldbaum M., Cai W. (2018). Identifying medical diagnoses and treatable diseases by image-based deep learning. *Cell*.

[3] Lee J. (2020). Integration of digital twin and deep learning in cyber-physical systems: towards. *Smart Manufacturing*.

[4] O’Shea T., Hoydis J. (2017). An introduction to deep learning for the physical layer. *IEEE Transactions on Cognitive Communications and Networking*.

[5] Ravi D., Wong C., Deligianni F. (2017). Deep learning for health informatics. *IEEE Journal of Biomedical and Health Informatics*.

[6] Schirrmeister R. T., Springenberg J. T., Fiederer L. D. J. (2017). Deep learning with convolutional neural networks for EEG decoding and visualization. *Human Brain Mapping*.

[7] Weilong Hou W., Xinbo Gao X., Dacheng Tao D., Xuelong Li (2015). Blind image quality assessment via deep learning. *IEEE Transactions on Neural Networks and Learning Systems*.

[8] Li X., Wang Y., Cai Y. (2021). Automatic annotation algorithm of medical radiological images using convolutional neural network. *Pattern Recognition Letters*.

[9] Wang X., Gao L., Mao S. (2016). CSI phase fingerprinting for indoor localization with a deep learning approach. *IEEE Internet of Things Journal*.

[10] Young T., Hazarika D., Poria S., Cambria E. (2018). Recent trends in deep learning based natural language processing [review article]. *IEEE Computational Intelligence Magazine*.

[11] Abdulazeez A. M. (2021). Electrocardiogram classification based on deep convolutional neural networks: a review. *Fusion: Practice and Applications*.

[12] Goh G. B., Hodas N. O., Vishnu A. (2017). Deep learning for computational chemistry. *Journal of Computational Chemistry*.

[13] Kumud S., Shruti A. (2021). A hybrid approach for neural network in pattern storage, fusion. *Practice and Applications*.

[14] Liu X., Li Y., Wang Q. (2018). Multi-view hierarchical bidirectional recurrent neural network for depth video sequence based action recognition. *International Journal of Pattern Recognition and Artificial Intelligence*.

[15] Sandberg J., Barnard Y. (2018). How can deep learning advance computational modeling of sensory information processing?.

[16] Lee J. G., Jun S., Cho Y. W. (2017). Deep learning in medical imaging: general overview. *Korean Journal of Radiology*.

[17] Yu D., Li J. (2017). Recent progresses in deep learning based acoustic models. *IEEE/CAA Journal of Automatica Sinica*.

[18] Lei X. (2021). Construction Technology and Quality Control of Power and Electrical Engineering Based on Convolutional Neural Network. *Security and Communication Networks*.

[19] Ye J., Ni J., Yi Y. (2017). Deep learning hierarchical representations for image steganalysis. *IEEE Transactions on Information Forensics and Security*.

[20] Zhao Z., Chen W., Wu X., Chen P. C. Y., Liu J. (2017). LSTM network: a deep learning approach for short‐term traffic forecast. *IET Intelligent Transport Systems*.

[21] Li H., Ota K., Dong M. (2018). Learning IoT in edge: deep learning for the internet of things with edge computing. *IEEE Network*.

[22] Han J., Zhang D., Cheng G., Liu N., Xu D. (2018). Advanced deep-learning techniques for salient and category-specific object detection: a survey. *IEEE Signal Processing Magazine*.

